RETRACTED

# Diagnosis of Breast Cancer Pathology on the Wisconsin Dataset with the Help of Data Mining Classification and Clustering Techniques

**DOI:** 10.1155/2022/6187275

**Published:** 2022-04-01

**Authors:** Walid Theib Mohammad, Ronza Teete, Heyam Al-Aaraj, Yousef Saleh Yousef Rubbai, Majd Mowafaq Arabyat

**Affiliations:** ^1^Al-Hussein Bin Talal University, Princess Aisha Bint Al Hussein College for Nursing and Health Sciences, Jordan; ^2^Al-Hussein Bin Talal University, Princess Aisha College for Nursing and Allied Science, Nursing Department, Jordan; ^3^Al-Hussein Bin Talal University, Princess Aisha Bint Al-Hussein College of Nursing and Health Sciences, Ma'an, Jordan; ^4^University of Petra, Jordan University of Science and Technology, Jordan

## Abstract

Breast cancer must be addressed by a multidisciplinary team aiming at the patient's comprehensive treatment. Recent advances in science make it possible to evaluate tumor staging and point out the specific treatment. However, these advances must be combined with the availability of resources and the easy operability of the technique. This study is aimed at distinguishing and classifying benign and malignant cells, which are tumor types, from the data on the Wisconsin Diagnostic Breast Cancer (WDBC) dataset by applying data mining classification and clustering techniques with the help of the Weka tool. In addition, various algorithms and techniques used in data mining were measured with success percentages, and the most successful ones on the dataset were determined and compared with each other.

## 1. Introduction

The quantity and variety of data have expanded in full agreement with the number of measurement tools in recent years. Massive amounts of data must be stored and analyzed in data warehouses due to developments in data collection methods and database technology. The process of finding the information hidden in the data obtained from many sources is called data mining [1]. Many open source and commercial programs are used to perform these operations. Open-source programs include WEKA, ARTool, RapidMiner, C4.5, etc. [2].

There are many studies conducted with WEKA, an open-source data-mining program in the literature. There are studies such as diagnosis and prediction of breast cancer cells [3], diagnosis and prediction of breast cancer [4], and diagnosis and prediction of Parkinson's disease. Only in the “IEEE Xplore” and “ScienceDirect” database searches with the keyword “WEKA,” there are 144 academic studies for the first and 1415 articles, 88 books, and 6 reference studies for the other.

It is the diagnosis of breast cancer 1, which has the highest incidence globally after breast cancer, by applying various data mining and machine learning techniques on data obtained from people diagnosed with this disease [4]. The contribution of study is distinguished and classifies benign and malignant cells, which are tumor types.

RETRACTED

### 1.1. Breast Cancer

Breast cancer is one of the most common diseases in women aged 40 to 59 years with multiple associated risk factors: genetic, environmental and behavioral factors, characterized by the disordered proliferation and constant growth of cells in this organ. Inflammatory breast cancer is rare and usually presents aggressively, compromising the entire breast, leaving it swollen and hyperemic [5, 6]. The initial symptomatology is a small nodule in the breast, usually painless and can grow slowly or quickly depending on its carcinogenesis. It must be approximately one centimeter in diameter for breast cancer to become palpable. And it takes years for it to reach this size, so early diagnosis is even more difficult, as eighty percent of cancers manifest as painless tumors, where only a minority, 10% of patients complain of pain without the perception of the tumor. There is a wide variation in the clinical course of breast cancer, as well as the length of time that patients can expect to live. An array of still-unknown mechanisms, such as the patient's immune, hormonal, and nutritional condition, influences this variance, such as the difference in tumour duplication speed and tumour metastatic potential.

Whether a tumor is benign or malignant is determined by pathological examination.

Benign tumors can be removed surgically and do not reappear. Most importantly, as we mentioned above, benign tumor cells do not invade other tissues and do not spread to other parts of the body. In other words, these tumors are not life-threatening.

Cancerous tumours are those that have undergone a malignant transformation. There is an uncontrolled proliferation of cancer cells. However, they grow and multiply far more quickly than benign tumors. They enter the body and cause harm to the nearby tissues and organs. Even if a tumor is malignant, cancer cells can escape from it and travel through the bloodstream or lymphatic system. Cancerous tumors, such as those found in the breast and elsewhere, develop in this manner.

When a tumor grows in the breast, it is known as breast cancer. Second, only to lung cancer, breast cancer is the most common cancer globally in terms of incidence. Breast cancer is estimated to affect one in eight women at some point in their lives [7]. Even though men can be affected, women are 100 times more likely than men to be affected. The modern, Western lifestyle is to blame for a rise in breast cancer incidence during the 1970s. More people in North America and Europe are affected by it than any other region. If breast cancer is detected early, the patient has a 96% chance of survival before it spreads. One woman in 44000 dies from breast cancer each year. The best preventive method against breast cancer is early detection. There is only one way to know whether the mass in the breast is benign (benign) or malignant (malignant). But some features can give an average idea to the examining physician about what that mass looks like [7].

RETRACTED

## 2. Experimental Study

One of the best examples that can be given to applying certain techniques to medical studies is the diagnosis of cancer and various diseases, as the advances in computer technologies and the field of computer science such as bioinformatics carry the developments in information technologies to the medical world. In line with the studies on this subject, we tried to determine breast cancer by working on the data in breast cells with data mining methods in our project. At this point, the Wisconsin Diagnostic Breast Cancer (WDBC) dataset created in cooperation with the University of Wisconsin and Madison Clinical Sciences Center was used as the dataset, and the Waikato Environment for Knowledge Analysis (Weka) tool developed by the University of Waikato was used as the classification and clustering tool.

### 2.1. Characteristics of the Dataset Used

Our dataset was obtained by imaging a needle-tip-wide breast mass with biosip by Dr. William Wolberg, an employee of Wisconsin Hospital, and digitizing these images by William Nick Street, one of the researchers of the University of Wisconsin Computer Sciences Department, in November 1995 [8]. In Figures 1 and 2, the images that make up our dataset are the originals.

Our dataset consists of a total of 569 samples. There are a total of 32 features that characterize our samples, the first of which is the ID of the sample, the second is its class, and the remaining 30 are features that contain various information about the cells. The class label of our samples can be malignant (M) or benign (B). These are medical terms that refer to the benign and malignant tumor cells we talked about earlier. There are no missing values for the properties. Of our samples, 357 are benign and it is distributed to be 212 malignant. Thanks to the 10-fold cross-validation classifier correctly created on our data, the classification success increased to a value of 97.5%. It correctly classified the 176 patients who came before November 1995 [9].

In Table 1, various features of our data are given together with their original form.

### 2.2. Techniques and Classifiers Used in the Experiment

This study's primary challenge is determining whether or not an unknown tissue sample is malignant or noncancerous. Multicategory categorization techniques are available in the literature. Five of these algorithms were chosen. Their classification capabilities were assessed on the relevant data set, based on their widespread use in biological sciences investigations and their proven success in other domains. C4.5 Decision Tree (DT), Artificial Neural Networks (ANN), Support Vector Machines (SVM), Naive Bayes multinomial classifier (NBM), and *K*-nearest neighbors (KNN) are some of the algorithms used (KNN) [10, 11].

RETRACTED

#### 2.2.1. Bayesian Classifier

In a classification problem, a simple classification form called “Naive Bayes” has emerged, based on conditional probability, assuming that the contribution of all features to the classification is equal and independent from each other. Accordingly, a conditional probability value is determined by analyzing the contribution of each independent feature to the result. Classification is performed by combining the effects of different attributes on the result. This method is called “naive” because the assumption that different attributes are independent of each other. The probability that the *t*_*i*_ record associated with a given data value *x*_*i*_ will be found in class *C*_*j*_ which is shown as *P*(*C*_*j*_ | *x*_*i*_). The training data can be used to calculate probabilities *P*(*x*_*i*_), *P*(*x*_*i*_ | *C*_*j*_) and *P*(*C*_*j*_). From these values, the posterior probabilities of *P*(*C*_*j*_ | *x*_*i*_) and then *P*(*C*_*j*_ | *t*_*i*_) are calculated by Bayes' theorem [12, 13].

To categorise a record, the training dataset is used to calculate conditional and a priori probabilities. When all of these attributes are taken into account, a total effect may be determined. There are several advantages to the “Naive Bayes” method. To begin with, it is quite simple to use. Second, unlike most other classification algorithms, only a single scan of the training data is required to achieve classification accuracy. Probability calculations can also be simplified by omitting blank values. As a general rule, it works well in circumstances where there are few or no complex relationships.

“Naive Bayes,” despite its ease of use, may not always yield good results. To begin with, it is possible that qualities are not mutually exclusive. Feature subsets can be employed in this situation. Second, this method is unable to deal with values that are not discrete. Intervals are needed to break up the continuous data. In addition to these issues, although there are associated answers, these solutions are difficult to implement, and the way these solutions are applied has a significant impact on the outcomes. Below is the classification study data created by applying the Naive Bayes technique with 10 selected, the most used *k*-fold cross validation value, to our dataset. Accordingly, the success rate and complexity matrix of the technique are as follows:

The values that mean the most to us here are the first two values. In other words, the number of samples classified correctly and incorrectly by the classifier and their percentages. As seen in Figure 3, the success rate of this method is 92.97%, and 529 out of 569 samples were classified correctly. However, the complexity matrix also contains very important information in measuring the system's success. The complexity matrix created by the Naive Bayes technique on this dataset is given in Table 2.

RETRACTED

Likewise, meaningful information such as TP, FP, and *F*-measure was formed as shown in Figure 4.

The success percentage of the applied method does not always give precise information about that method. In addition to the success rate, measurements such as the accuracy rate (TP rate) and the misclassification rate (FP Rate) provide very important information for the system's success because the meaning of these numerical values is very great in the processes where the diagnosis of cancer is very serious.

#### 2.2.2. Neural Network-Based Classifiers [14]

When they are used, a model is created to output the probabilities of a given sample being in the current classes. When this model is applied, the output that gives the highest value is considered the result class. In the training phase, when each data is given into the artificial neural network, the weight values in the network change based on the comparison of the result with the expected result. Classification problem with the neural network consists of the following steps:

1. Determining the attributes for the input and the number of outputs
2. Determining the number of hidden layers and the number of hidden nodes in the hidden layers depending on the relevant problem area
3. Determining the weights and functions to be used in the network
4. Determination of the training dataset. Too much training data can cause “overfitting,” and too little training data can cause “underfitting”
5. Determination of the learning technique. This technique determines how the weights are arranged. Mostly, an approach in the form of backpropagation is followed
6. Determination of the stopping condition. The learning process can be terminated when all the training data are evaluated on the network or when a desired error rate or a specified time criterion is reached
7. They are comparing the result with the desired result by evaluating each training data in the network until the stopping condition is met. If the result is as desired, adjusting the weights increases the probability of getting the same result when similar data is received. If the result is different from the desired, weight changes are made to reduce the probability of this result being repeated
8. Classification of the data to be tested due to the evaluation in the trained network

This time, our dataset will be classified with the multilayer perceptron classifier of artificial neural networks and the results will be evaluated according to this method in Table 3. This method is available under the name multilayer perceptron in the Weka tool as shown in Figure 5.

RETRACTED

As shown in Figure 6, compared to the Naive Bayes technique, the multilayer perceptron technique achieved higher results of incorrect classification of benign and malignant cells. Therefore, it is more successful in this dataset compared to the Naive Bayes classifier.

#### 2.2.3. Support Vector Machines (SVM)

SVM is a privileged classifier defined by hyperplanes that divide the problem space into various parts. [15] In other words, it is an algorithm for finding the optimum hyperplanes that separate a given training data set and the relevant data as a result of supervised learning. What is the optimal hyperplane is the main factor that creates the privilege of SVM and determines the classification performance in Table 4.

In the Weka tool, this method is called the SVM technique. The output information generated by this technique is shown in Figure 7.

As shown in Figure 8, the point that draws attention here is that the number of samples correctly classified by the technique is the same as the previous multilayer perceptron technique for malignant cells, but the success of classifying benign cells is more successful than the multilayer perceptron technique. Therefore, the number and percentage of correctly classified samples are more successful than those of the previous method.

#### 2.2.4. Decision Tree Classifier (J48)

The basis of classification with the decision trees approach is to divide the search space into rectangular regions [16, 17]. The record to be evaluated will be classified according to its region. Although there are some different approaches, a decision tree can be defined as follows: In a data set given as *D* = {*t*_1_, ⋯, *t*_*n*_}, let the record be *t*_1_ = <*t*_*i*1_, ⋯, *t*_*ih*_> and the records {*A*_1_, ⋯, *A*_*h*_} attributes. Classes of related records are also *C* = {*C*_1_, ⋯.Let it be *C*_*m*_ }. In this case, a decision tree associated with *D* should have the following properties:

- The root node and each intermediate node must be defined with an attribute
- Each branch should represent a value or range of values of the attribute at its starting point
- Each leaf node must be represented as a *C*_*j*_ class

In this case, each different path starting from the root node to a leaf node defines a rule consisting of “AND” operations. When these rules are applied to any data, only one of the rules will terminate successfully. The classification result is the leaf node value in the path that creates this rule.

RETRACTED

There are important points to be determined in the decision trees, such as finding the attributes used in the root and intermediate nodes and which value ranges of these attributes will be used. The general principle in decision trees is to find the attributes that sequentially divide the training data into different classes in the best way and to find the value ranges at the nodes where these attributes will be applied to the data set. These selected attributes can be called distinctive attributes as shown in Table 5.

Decision trees are available in the Weka tool with many different methods. The most used ones are the ID3 algorithm and the J48 technique. For our dataset, the ID3 algorithm is turned off in Weka. Therefore, we apply the J48 technique and find the results as shown in Figure 9.

As can be seen from the results, the J48 technique is a more unsuccessful method compared to all other methods, except for the Naive Bayes classifier as shown in Figure 10.

#### 2.2.5. *K*-Nearest Neighbor (KNN)

One of the supervised learning strategies for solving the classification problem is the *K*-nearest neighbor method [18, 19]. By assessing the similarity of the data to be classified in the technique to the normal behavior data in the learning set, they are assigned to the classes based on the specified threshold value. The crucial thing is that each class's attributes are predetermined. The number of *k*-nearest neighbours, the threshold value, the similarity measurement, and a sufficient number of normal behaviours in the learning set all influence the method's performance. In Table 6, on Weka, the *K*-nearest neighbour approach is known as KNN. The following is the classification result obtained using the KNN algorithm as shown in Figure 11.

### 2.3. Clustering Methods Used in the Experiment

As shown in Figure 12, as the name suggests, the practice of organising data into clusters is known as clustering. A “cluster” is the collective term for each of these collections. Cluster analysis, or “clustering,” is a shorthand term for this type of study. The elements inside a cluster should have a high degree of similarity, and the clusters should have a low degree of similarity. Unattended classification, or clustering, is the next step in evolving data mining techniques. The goal of unsupervised classification is to organize the data into meaningful subsets for a given collection of data. In this dataset, we used two kinds of clustering techniques. Both *K*-means and hierarchical clustering can find these patterns in the data set.

RETRACTED

#### 2.3.1. *K*-Means Clustering

The two most preferred methods in the nonhierarchical clustering method are the *k*-means technique developed by Mac Queen and the maximum likelihood technique [20, 21] as indicated in Table 7. In this study, an application of nonhierarchical clustering algorithms has been developed. The results of this method are given in Figure 13.

#### 2.3.2. Hierarchical Clustering

In the hierarchical clustering method, the dendrogram (tree graph) is used to make the operation easier to understand [22]. The most used hierarchical methods based on the operations described in the hierarchical clustering method are single link, full link, average link, central, and ward methods. In Table 8, the nonhierarchical clustering method, on the other hand, is preferred if there is prior knowledge about the number of clusters or if the researcher has decided on the number of clusters that will be meaningful. The results of this method are given in Figure 14.

## 3. Conclusion

As a result, J48 and *K*-nearest neighbor (KNN) from Naive Bayes, decision support machine (SVM), multilayer perceptron (MLP), and decision tree methods, which are the five most used classifier techniques, were applied on our dataset, and the highest success rate was 97.7% percent; it belongs to the decision support machine method. This method was followed by multilayer perceptron, KNN, J48 decision tree, and Naive Bayes. From these results, we understand that using the SVM technique while classifying our dataset will achieve more successful results in classifying tumor cells correctly. A graphical representation (Figure 15) of these methods' percentages and accuracy rates is given.

## Figures and Tables

**Figure 1:** Image of a benign tumor cell.

**Figure 2:** Image of a malignant tumor cell.

**Figure 3:** Data of the Naive Bayes technique.

**Figure 4:** Accuracy and sensitivity information of the Naive Bayes technique.

**Figure 5:** Success percentages of the multilayer perceptron technique.

**Figure 6:** Accuracy and sensitivity information of the multilayer perceptron technique.

**Figure 7:** Success percentages of the SVM technique.

**Figure 8:** Accuracy and sensitivity information of the SVM technique.

**Figure 9:** Success percentages of the J48 technique.

RETRACTED

**Figure 10:** Accuracy and sensitivity information of the J48 technique.

**Figure 11:** Percentages of success of the KNN technique.

**Figure 12:** Accuracy and sensitivity information of the KNN technique.

**Figure 13:** Success percentages of the *K*-means technique.

**Figure 14:** Success percentages of the hierarchical clustering technique.

**Figure 15:** Comparison of classifiers.

**Table 1:** Characteristics of the samples.

(i) Radius: radius of all cells are shown by the mean, standard deviation, and worst value
(ii) Texture: the mean, standard deviation, and worst value of the grayscale change rates of interior surfaces are shown in the table below.
(iii) Perimeter: the perimeters of the cells were measured for the mean, standard deviation, and worst value
(iv) Area: the mean, standard deviation, and worst-case value of the surface areas of the cells are all calculated and displayed
(v) SVMothness: The average, standard deviation, and worst value of the radius lengths of neighbouring cells are all displayed in the graph (vi) Compactness: perimeter^2^/area = density mean, standard deviation, and worst value
(vii) Concavity: the mean, standard deviation, and worst value of the indentations and protrusions around the cell are all displayed on this graph
(viii) Concave points: the mean, standard deviation, and worst value for the number of indentation and protrusion sites around the cell are all calculated using this data
(ix) Symmetry: the mean, standard deviation, and worst value of the change in ellipse shape of cells were calculated
(x) Fractal dimension: there are three values for this ratio: the mean, standard deviation, and worst value. There are three values for this ratio.

**Table 2:** The complexity matrix of the Naive Bayes technique.

		Estimated value	
		Malignant	Benign
Actual value	Malignant	191	21
	Benign	16	341

**Table 3:** Complexity matrix of the multilayer perceptron technique.

		Estimated value	
		Malignant	Benign
Actual value	Malignant	200	10
	Benign	9	342

**Table 4:** Complexity matrix of the SVM technique.

		Estimated value	
		Malignant	Benign
Actual value	Malignant	200	10
	Benign	3	356

**Table 5:** Complexity matrix of the J48 technique.

		Estimated value	
		Malignant	Benign
Actual value	Malignant	195	17
	Benign	24	333

**Table 6:** Complexity matrix of the KNN technique.

		Estimated value	
		Malignant	Benign
Actual value	Malignant	199	13
	Benign	12	345

**Table 7:** Complexity matrix of the *K*-means technique.

		Estimated value	
		Malignant	Benign
Actual value	Malignant	179	31
	Benign	10	349

**Table 8:** Complexity matrix of the hierarchical clustering technique.

		Estimated value	
		Malignant	Benign
Actual value	Malignant	2	211
	Benign	0	356

RETRACTED

## Data Availability

The data used to support the findings of this study are included within the article.
